The article "The case of philanthropy: bringing scientists and philanthropic donors together, for good" was published in 2015. Journal: Dis Model Mech.

# The case of philanthropy: bringing scientists and philanthropic donors together, for good

**DOI:** 10.1242/dmm.022178

**Published:** 2015-09-01

**Authors:** Olivia Tournay Flatto

**Affiliations:** Olivia Tournay Flatto, PhD is the Co-Founder and Executive Director of the Pershing Square Sohn Research Alliance (PSSCRA). She also serves on the boards of The Pershing Square Foundation; The Public Good Projects; American Friends of the Paris Opera and Ballet (Chairman); Paris Opera and Ballet; and the New Leaders Group at the Institute of International Education (IIE). Pershing Square Sohn Research Alliance (PSSCRA), New York, NY 10019, USA

## Abstract

**Summary:** Philanthropists and scientists share many common interests, and yet they are not familiar with each other's ways of thinking. This Editorial highlights how to improve their mutual understanding to advance research and life sciences.

“Wealth is not new. Neither is charity. But the idea of using private wealth imaginatively, constructively, and systematically to attack the fundamental problems of mankind is new.” – John Gardner

Philanthropy, derived from private wealth, stands unique as a vital source of scientific funding. Yet many scientists don't truly understand the workings of this form of charitable giving. Some are even wary of it, and believe that a divide between the worlds of science and business is a normal state of affairs. My experience has exposed striking similarities between the two specialties: both dedicate their resources to innovation and the sincere desire to do good for their fellow man.

I've been lucky to work on both sides of the fence. I conducted research for my PhD at the Wistar Institute in Philadelphia, PA, and at Sloan Kettering Institute in New York City, NY, where I worked on the *Id1* gene and its role in the molecular mechanism of mammalian cell differentiation. I later moved to the Pershing Square Foundation. In 2013, to support young investigators with bold and risky ideas in cancer research in the New York area, the Pershing Square Foundation partnered with the Sohn Conference Foundation to create the Pershing Square Sohn Research Alliance (PSSCRA). Since the organization's founding, I have served as its Executive Director. As a result of my career experience, I understand firsthand the role of philanthropic support of medical research. I am always excited to work with new, young and innovative talent, and to introduce that talent into the social mainstream.

## Philanthropy today: measuring impact

Philanthropy, like everything in this high-tech world, has changed dramatically in the past few years. There was a time when donors did not focus on measuring the impact of their gifts. Only a few individuals were wealthy enough to establish foundations and provide funds to build museums, programs and art collections. In today's world, foundations strive to be part of the scientific solution, to provide money that goes to new advancements, such as the discovery of a new molecule. Of course, present-day donors have become increasingly more sophisticated in their expectations and want to see a return on their investment. They have a clear picture of the issues, and foundations and donors want to measure their impact.

The article "The case of philanthropy: bringing scientists and philanthropic donors together, for good" was published in 2015. Journal: Dis Model Mech.

One important way to measure impact is by observing whether the project scales up and leverages additional types of funding. More than ever, donors think in terms of business-model philanthropy when considering social investments. This model is not incompatible with that of science; the short-term goal of funding new basic discoveries is consistent with the long-term goal of a financial return stemming out of the commercialization of a new drug.

## Philanthropy touts innovation and rewards risk

Philanthropists give money generously for a variety of reasons. Some examples include: **The Civic-Minded Donor** who seeks to help the community. He or she seeks out worthy causes and donates to them; **The Foundation Donor** has the money to start his or her own foundation, usually with specific interests in mind – health, social entrepreneurship, poverty or the environment; **The Donor with a Cause** raises money for a specific purpose. The Michael J. Fox Foundation for Parkinson's Research, and The Breast Cancer Research Foundation are prime cases.

All these philanthropists are viable funding sources for scientific researchers. They offer dynamic alternatives to traditional resources. Although the United States is well known for having many private philanthropists (in my native France, by contrast, research funding is provided almost exclusively by the government), it functions under economic constraints that make private philanthropic money even more crucial. Philanthropy will not replace what the government does but, by its nature, can do things the government can't or won't. Bold, innovative projects need funding at the earliest stages.

The National Institutes of Health (NIH), the United States' preeminent public source of scientific research funding, is traditionally risk-averse and regularly funds only incremental research. Budgeted at $30-billion per year, the NIH has, for the past 10 years, received no increase in its budget, and has had funding cut through sequestration. Consequently, it finances and rewards safe and predictable projects.

Conversely, foundations in medical research can fill a unique niche by supporting new and risky projects early on, understanding that the investment is more long-term.

The article "The case of philanthropy: bringing scientists and philanthropic donors together, for good" was published in 2015. Journal: Dis Model Mech.

Philanthropists and programs like the PSSCRA, are willing to identify the ‘budding’ scientist, the up-and-comer. In short, investing in the future leaders of the next generation.

## Scientists should take risks: changing perceptions

The nature of scientific work requires solitude and isolation. Researchers work methodically, with great concentration. Their single-mindedness and sensitivity suit them well for exploration into molecular frontiers and, as a result, they are less exposed to the business and philanthropic worlds in the early stages of their career. In addition, the perceived dissimilarity between the worlds of science and business has for a long time led many researchers to hold a lingering skepticism of commerce. The need to collaborate and the changes in the funding landscape have altered this perception.

The scientist has many factors to consider when approaching funding sources. First, the NIH rewards safety and predictability. Knowing this, the scientist is often inhibited from submitting risky projects to the NIH. Next, scientists are rewarded by the quality and amount of publication. A risky project financed primarily by foundations, for example, is less likely to turn into a paper in the foreseeable future, which presents challenges to the traditional model of advancement and also inhibits the type of research that is done.

## How to bridge the gap

It is imperative that we create other funding paths for scientists that enable them to push forward their boldest research. By creating the PSSCRA (‘the Alliance’), we are seeking to bridge the gap between scientists and the business and philanthropic communities in New York. We made it our mission to bring them together so that today's scientists can take the risks needed to find the solutions for tomorrow.

The Alliance is based in New York City, which is a special place. So much talent is concentrated in such a little area, spanning many disciplines, the arts and business. Where but in New York City can the entrepreneur sit beside the artist, the scientist beside the captain of industry?

Leveraging the Alliance's events, which are incredibly focused networking opportunities, the Alliance brings together scientists, leaders in industry, heads of large foundations and business community leaders. We take pride in creating these vibrant mentoring relationships and connections.

Building communities and networks around the scientists is one of the elements of success that we have identified as being crucial to their growth and exposure. Each one of our Prize Winners is paired with a mentor in the pharma or biotech industries. Thus, the three important pillars of our program are: (1) the selection of the scientists, (2) their match with a mentor, and (3) measuring the impact of this program. Ultimately, there's nothing better than validation, and the new-model foundation offers it both professionally and socially.

The article "The case of philanthropy: bringing scientists and philanthropic donors together, for good" was published in 2015. Journal: Dis Model Mech.

## Finding talented scientists

“To give away money is an easy matter and in any man's power. But to decide to whom to give it and how large and when, and for what purpose and how, is neither in every man's power nor an easy matter.” – Aristotle

When we instituted the Pershing Square Sohn Prize for Young Investigators in Cancer Research (now in its second year), the search began by reaching out to all the communication and development offices of every scientific research institution and university department in the New York area, placing banner ads in the most prominent and interesting scientific magazines, and sending personalized emails to chairs, heads of departments and individual scientists. “Spread the word,” we told them.

Ads in special-interest magazines and websites for specific groups are important. Even though our search is broad, this puts us on very specialized radars.

Every institution has a grant department, individual gift department or foundation organization that assesses needs and suggests funding options. We wanted to encourage each scientist who has an innovative idea to apply. We wanted a democratic process. And, even if they have funding for another area of their research, they might not have it for the innovative, risky idea.

In the first year, we received 64 applications. This year, we received 67 applications. We look at the quality of each applicant, the project's innovative approach and its relevance in cancer research. After a first round of screening last year, we asked 28 applicants to return for full submission.

After the submission process, each application is reviewed by three experts in the field. The finalists present their work in a boardroom where the leaders in the field are present. This is unique exposure for our young innovators. Finally, we chose six Prize Winners in 2014 and another six in 2015.

The Prize Winners are then invited for individual meetings with a mentor in the pharmaceutical or biotech company. Mentors are exposed to research that they would not be otherwise. It's a way for pharma and academia to exchange ideas and build on each other’s strengths.

For philanthropists, there is nothing more satisfying than to have personal contact with the individuals whom they are helping and to understand their needs better so that they can be more effective. Philanthropy is uniquely positioned to take risks. We want to identify future innovators. And so, our relationship to a grantee is very important. Non-profit organizations that raise money and do not give donors direct access to see what their money is doing are going to lose them. It's satisfying to fund the future musical genius…why not the future Nobel Prize Winner? And, young scientists are excited to know they're part of that prestigious group.

The article "The case of philanthropy: bringing scientists and philanthropic donors together, for good" was published in 2015. Journal: Dis Model Mech.

Times are changing. Technology has brought us closer and piqued our interest in all facets of life. Science and philanthropy are changing as well and share the common goal of providing our society with enlightenment. Now is the perfect time to bring these two attributes together.

